RETRACTED

# Deployment optimization of multi-stage investment portfolio service and hybrid intelligent algorithm under edge computing

**DOI:** 10.1371/journal.pone.0252244

**Published:** 2021-06-04

**Authors:** Xuecong Zhang, Haolang Shen, Zhihan Lv

**Affiliations:** 1 College of Information Science and Technology, Jinan University, Guangzhou, China; 2 Jinan University- University of Birmingham Joint Institute, Jinan University, Guangzhou, China; 3 School of Data Science and Software Engineering, Qingdao University, Qingdao, China; Ministry of Natural Resources North Sea Bureau, CHINA

## Abstract

The purposes are to improve the server deployment capability under Mobile Edge Computing (MEC), reduce the time delay and energy consumption of terminals during task execution, and improve user service quality. After the server deployment problems under traditional edge computing are analyzed and researched, a task resource allocation model based on multi-stage is proposed to solve the communication problem between different supporting devices. This model establishes a combined task resource allocation and task offloading method and optimizes server execution by utilizing the time delay and energy consumption required for task execution and comprehensively considering the restriction processes of task offloading, partition, and transmission. For the MEC process that supports dense networks, a multi-hybrid intelligent algorithm based on energy consumption optimization is proposed. The algorithm converts the original problem into a power allocation problem via a heuristic model. Simultaneously, it determines the appropriate allocation strategy through distributed planning, duality, and upper bound replacement. Results demonstrate that the proposed multi-stage combination-based service deployment optimization model can solve the problem of minimizing the maximum task execution energy consumption combined with task offloading and resource allocation effectively. The algorithm has good performance in handling user fairness and the worst-case task execution energy consumption. The proposed hybrid intelligent algorithm can partition tasks into task offloading sub-problems and resource allocation sub-problems, meeting the user’s task execution needs. A comparison with the latest algorithm also verifies the model’s performance and effectiveness. The above results can provide a theoretical basis and some practical ideas for server deployment and applications under MEC.

## 1. Introduction

With the advent of smart cities and the Fifth Generation (5G) technology, the Internet of Things (IoT) technology is developed quickly, and loads of data are generated [1]. In recent years, portable devices, such as mobile phones, tablets, and notebooks, have occupied most people’s daily lives due to their convenience. More devices are connected to the internet and generate data. According to statistics, by 2020, each person will generate an average of 1.5GB of data per day [2]. However, it is difficult for mobile devices to process these data. For example, facial recognition, natural language processing, and virtual reality have no suitable applications on traditional devices [3]. Second, many technologies are challenging to implement on mobile devices due to the limitations of devices’ battery life, computing power, and size [4]. Mobile cloud computing has been widely applied to overcome the above obstacles, whose foremost idea is to offload computationally intensive tasks that require a large number of computing resources in mobile devices to remote clouds instead of executing locally [5]. Mobile Edge Computing (MEC) allows terminal devices to offload computationally intensive tasks to mobile edge servers for execution. The mobile edge servers with high computing performance can reduce the task execution time delay [6]. In the meantime, because the terminal offloads its computing tasks, the energy consumption required to perform tasks can be significantly reduced. Therefore, the mobile edge can effectively alleviate the principal contradiction between smart terminals’ resource limitation and high-performance task processing demand [7]. Although mobile cloud computing has apparent advantages in solving the above problems, the distance between the cloud server and the user increases the delay. This cloud computing cannot meet the needs of 5G network users. Also, loads of mobile devices connected to the cloud and competing for resources will cause severe network congestion, severely hindering the industry’s development [8]. Therefore, studying the server deployment problem under MEC has significant practical value for the IoT industry’s development.

RETRACTED

With the development of the mobile internet and the popularization of smart terminals, various new applications, such as augmented reality, virtual reality, and natural language processing, continue to emerge [9]. These applications usually have resource-intensive characteristics and require many computing resources and storage resources when running, affecting service quality. Although smart terminal processors’ performance continues to increase, they cannot process high-performance applications in a short time, seriously impacting the user’s service experience [10]. Therefore, how to expand intelligent terminal resources to meet the needs of high-performance task execution is an urgent problem that needs solving. Many scholars have researched MEC. Huang et al. (2019) proposed a system model for multi-user mobile task offloading. They studied the placement of server deployment and the impact of mobile users on network allocation. They designed an algorithm to solve this problem, aiming to place servers in areas with high user density and assign mobile users to different locations. The final experiment proved the effectiveness of the algorithm [11]. Jiang et al. (2020) investigated cloud servers’ layout using multiple wireless access points and formulated the problem as a new capacity-based cloudlet layout problem, which placed K servers in different strategic locations. A practical solution was designed to minimize the access delay between mobile users and the servers serving the users [12]. Li et al. (2021) explored the offloading of multi-user computing in mobile edge computing in a multi-channel wireless interference environment. They expressed the decision-making problem of distributed computing offloading among mobile device users as a multi-user computing offloading game and designed a distributed computing offloading algorithm to achieve Nash equilibrium [13]. According to the above works, there are many studies on MEC but less analysis of servers’ deployment. However, the latter plays a very crucial role in improving the transmission efficiency of IoT.

Given the above problems, a multi-stage-based task resource allocation model is proposed based on the traditional MEC for different resource allocation problems. This model comprehensively considers constraints such as task offloading, task partition, transmission rate, and resource allocation. It models the combined task offloading and resource allocation problems to solve task execution overhead minimization. A multi-hybrid intelligent algorithm based on energy consumption optimization is proposed for the MEC process supporting dense networks. This algorithm converts the original problem into task offloading sub-problems and resource allocation sub-problems, thereby determining the combined task offloading and resource allocation optimization strategies.

The purposes are to improve the efficiency of service deployment under mobile edge computing. The densely networked cellular MEC system is used as the research object, and a joint task offloading, and resource allocation algorithm is proposed based on energy consumption optimization. The maximum task execution energy consumption is defined as the maximum energy consumption required for each user’s task execution. Moreover, the constraints of task offloading, power allocation, transmission rate, and computing resource allocation are considered comprehensively. The joint task offloading and resource allocation problem is modeled as minimizing the maximum energy consumption of task execution, thereby determining the joint task offloading and resource allocation strategies.

RETRACTED

## 2. Methods

### 2.1 MEC framework

Fig 1 displays the MEC architecture released by ETSI. From a macroscopic perspective, this architecture divides the MEC platform into three levels according to the different partitions that implement functions. From top to bottom are the mobile edge system, the mobile edge host, and the network. The mobile edge system at the top is responsible for the overall management of the mobile edge system. It abstracts the system as an interface for users and third-party developers [14]. The mobile edge host in the middle is composed of mobile edge hosts and mobile edge host-level management. It is the core component of the MEC three-layer architecture. The mobile edge host provides a virtualized infrastructure and a mobile edge platform for mobile applications and is uniformly configured by the mobile edge host-level management. The bottom network supports multiple access methods for the platform and manages the access of the third-generation partner project cellular network, local area network, and other non-mobile networks [15].

**Fig 1:** A schematic diagram of the MEC framework.

Fig 2 shows the MEC reference architecture. The architecture focuses on refining the mobile edge system and the mobile edge host and defines functional entity interfaces to accomplish the signaling interaction between each functional entity. The primary interfaces include the mobile edge platform’s function correlation interface, the interface between managers, and interfaces connected with external entities [16].

**Fig 2:** A schematic diagram of MEC reference architecture.

### 2.2 Multi-investment portfolio and server deployment

A cellular MEC system supporting D2D communication consisting of a single base station with a MEC server deployed and multiple users is considered, as shown in Fig 3. Assuming that some users in the system need to perform computationally intensive tasks tolerated by the time delay, the MEC server deployed on the base station side can provide task offloading services for the server [17]. Therefore, in addition to perform the task locally, the server can also offload the task to the MEC server through the cellular link for execution. The task execution performance of all servers in the system is considered, and the task execution overhead is defined as:

$$U=\sum_{i=1}^{N}U_{i}$$ (1)

**Fig 3:** Multi-stage-based task resource allocation model.

In (1), *U*_*i*_ is the task execution overhead of *RU*_*i*_, where the task execution overhead of *RU*_*i*_ is modeled as:

$$U_{i}=x_{i}^{0}U_{i}^{0}+x_{i}^{b}U_{i}^{b}+\sum_{j=1}^{M}x_{i,j}^{d}U_{i,j}^{d}$$ (2)

In (2), $x_{i}^{0}$ represents the variable of the fully local execution mode, $x_{i}^{b}$ denotes the variable of the MEC offload execution mode, $x_{i,j}^{d}$ refers to the variable of D2D offload execution mode, $U_{i}^{0}$ stands for the overhead of the *RU*_*i*_ task with fully local execution, $U_{i,j}^{d}$ indicates the task offloading to the MEC server for execution overhead, and $U_{i}^{b}$ denotes the overhead for offloading task to *SU*_*j*_ execution. It is assumed that some users with strong computing power can provide D2D offloading services for their neighboring servers. Assuming that the tasks to be performed by the server can be partitioned into parts of any size, each part of the task can be executed in different modes in a parallel manner.

RETRACTED

Assuming that the server in the system can execute tasks using three modes: the fully local execution mode, the MEC offload execution mode, and the D2D offload execution mode. It is assumed that multiple servers can simultaneously access the base station to efficiently utilize the base station resources. Besides, it is assumed that multiple servers can offload their tasks to the MEC server through the cellular link simultaneously to fully utilize the MEC server’s computing power and improve the server’s task execution performance. Therefore, each server can be allocated a particular percentage of computing resources.

Here, the MATLAB simulation software is adopted to verify the performance of the proposed algorithm. The algorithm is then compared with the algorithm proposed in the literature [18] and the two baseline algorithms. The literature has studied some task offloading problems in the cellular network that supports MEC, modeled the combined task offloading and resource allocation problems to minimize the task execution time delay, and proposed an algorithm to solve the above problem effectively. The Optimal Resource Allocation (ORA) algorithm allocates bandwidth and computing resources to each server in an optimal manner, and the Equal Resource Allocation (ERA) algorithm allocates bandwidth and computing resources to each server in an equal manner [19].

The simulation scenario is a cellular D2D communication system supporting MEC composed of a base station, multiple servers, and multiple base stations. The simulation area is 1000m×1000m, and the servers and base stations are evenly distributed in the simulation area. The relevant parameters used in the simulation are shown in Table 1. The task input data volume, the number of computing resources required to complete the task, and the server’s computing power and the base station are randomly selected from Table 1 to describe the different requirements of the task and the different characteristics of the server the base station equipment. All simulation results are the average of 1000 independent simulations.

RETRACTED

**Table 1:** Simulation parameter determination of multi-stage investment portfolio server.

Parameter	Letter	Value	Parameter	Letter	Value
Base station bandwidth	*W*^*b*^	10 MHz	Sending power of the cellular link	*P*_*1*_^*b*^	600 mW
D2D link bandwidth	*W*^*d*^	5 MHz	Sending power of the D2D link	*P*_*1*_^*d*^	200 mW
Noise power	*ϭ*^*2*^	-75 dBm	Weight factor	*ρ*	0.01
MEC server’s computing power	*F*	30 Gcycles/s	Task input data volume	*I*_*i*_	[1, 2] Mbits
The number of computing resources required to complete the task	*D*_*i*_	[0.5, 0.6] Gcycles	The computing power of SU*j*	*F*_*j*_^*b*^	[1.2, 1.5] Gcycles/s
The computing power of Server *i*	*F*_*i*_	[0.8, 1] Gcycles/s			

### 2.3 Model construction and system settings

For cellular systems that support dense networking, user task characteristics, channel bandwidth differences between base stations, and mobile edge computing server available computing resources are comprehensively considered while noting the user fairness. A joint task offloading and resource allocation algorithm is proposed based on energy optimization. The specific structure is presented in Fig 4. The maximum task execution energy consumption is defined as the maximum energy consumption required for each user’s task execution. Under the constraints of task unloading, power allocation, transmission rate, and computing resource allocation, the joint task offloading and resource allocation problem is modeled as minimizing the maximum energy consumption of task execution. The task offloading and resource allocation can be jointly optimized by solving this problem.

**Fig 4:** The multi-hybrid intelligent algorithm based on energy consumption optimization.

(1) Objective function modeling: considering the fairness of users, the energy consumption of task execution is defined as the maximum energy consumption required for task execution of each user in the system, namely:

$$E=\underset{i\in \phi }{\text{max}}E_{i}$$ (3)

In (3), *E*_*i*_ denotes the task execution energy consumption of user *i*, where the task execution energy consumption of user *i* is modeled as:

$$E_{i}=(1-\sum_{j\in \varphi }x_{i,j})E_{i}^{0}+\sum_{j\in \varphi }x_{i,j}E_{i,j}$$ (4)

In (4), *x*_*i*,*j*_ represents the task offloading variable, $E_{i}^{0}$ denotes the local energy consumption of user *i*’s task, and *E*_*i*,*j*_ refers to the energy consumption required for offloading user *i*’s task to the small base station *j* and executing on its MEC server.

(2) Local execution mode: the local execution energy consumption of user *i*’s task is modeled as:

$$E_{i}^{0}=\sigma_{i}D_{i}F_{i}^{2}$$ (5)

In (5), *σ*_*i*_ represents the energy consumption coefficient associated with the user’s CPU performance, *D*_*i*_ denotes the computing resource required to complete the task of user *i*, and *F* describes the computing power of user *i*. MEC offloading execution mode: the task of user *i* is offloaded to small base station *j*, and the execution delay on its MEC server is modeled as:

$$E_{i,j}=E_{i,j}^{t}+E_{i,j}^{e}$$ (6)

In (6), $E_{i,j}^{t}$ represents the energy consumption required for user *i* to transmit task input data to small base station *j*, and $E_{i,j}^{e}$ represents the energy consumption required for user *i* to perform tasks on the MEC server of small base station *j*. Among them, the energy consumption required for user *i* to transmit task input data to small base station *j* is modeled as:

$$E_{i,j}^{t}=p_{i,j}T_{i,j}^{t}$$ (7)

In (7), *p*_*i*,*j*_ represents the power at which user *i* sends task input data to small base station *j*, and $T_{i,j}^{t}$ represents the delay required for user *i* to transmit task input data to small base station *j*. The time delay required for user *i* to transmit task input data to small base station *j* is modeled as:

$$T_{i,j}^{t}=\frac{I_{i}}{R_{i,j}}$$ (8)

In (8), *I*_*i*_ represents the amount of task input data for user *i*, and *R*_*i*,*j*_ represents the data rate at which user *i* transmits task input data to small base station *j*. The data rate at which user *i* transmits task input data to small cell *j* is modeled as:

$$R_{i,j}=W_{j}^{sub}\;{\text{log}}_{2}(1+\frac{p_{i,j}h_{i,j}}{\sigma^{2}})$$ (9)

In (9), $W_{j}^{sub}$ represents the sub-channel bandwidth of small base station *j*, *h*_*i*,*j*_ represents the transmission gain of user *i* and small base station *j*, and *σ*^*2*^ denotes the noise power of the transmission channel.

(3) Constraint modeling: the aims are to minimize the system’s maximum task execution energy consumption and design the optimal joint task offloading and resource allocation strategy. Therefore, the modeled optimization problem needs to meet the following constraints:

$$C1:\sum_{i\in \phi }x_{i,j}\leq \text{min}\{B_{j},S_{j}\}$$ (10)

In (10), *S*_*j*_ represents the maximum number of users served by the MEC server of the small base station *j*. The user’s transmission power is non-negative and should not exceed the maximum transmission power of the user. Regarding the limited computing resources of the MEC server, the sum of the resources allocated to each user should not exceed the MEC server’s total resources.

RETRACTED

Genetic Algorithm (GA) can start the search from the group and has potential parallelism. It can compare multiple individuals at the same time. The evaluation function inspires the search; the process is simple, and the probability mechanism is used for iteration, which is random. It has scalability and is easy to combine with other algorithms. The advantages of PSO are simplicity, easy implementation, no gradient information, and few parameters. In particular, its natural real-number coding characteristics are particularly suitable for real optimization problems. Ant Colony Optimization (ACO) has strong robustness and the ability to search for better solutions to solve performance compared with other heuristic algorithms. ACO is an evolutionary algorithm based on population, which is inherently parallel and easy to implement in parallel. In the mobile edge computing environment, edge servers’ placement can be regarded as a network, which is an undirected graph composed of many mobile users, many base stations, and a group of potential edge servers.

Regarding the insufficient initial pheromone in ACO, other algorithms are used to generate initial pheromone distribution, and ACO is used to find accurate solutions, thereby improving time efficiency and solution accuracy. In this regard, GA is introduced into each iteration process of ACO. The solution formed by each generation of the ant colony system is the initial population of other algorithms. Through multiple iterations of other algorithms, it tries to find a better solution, thereby speeding up the ant colony system’s convergence and increasing the solution rate. Usually, α and β in ACO are selected through experience, and improper selection will significantly reduce the performance of the algorithm. Therefore, other algorithms can train the ant colony system’s parameters α and β. Because ACO converges prematurely to the non-global optimal solution, and the time consumed is too long, ACO is used for searching. Then, other algorithms are used to search the effective routing path obtained by the ACO. After the optimization process of selection, crossover, and mutation, the performance will be improved, generating excellent next-generation groups.

Therefore, in addition to perform the task locally, the user can also offload the task to the MEC server through the cellular link for execution. The GA, Multi-particle Optimization (MPO) algorithm, and ACO are applied to form a fusion algorithm to deploy target resources to fully utilize the MEC server’s computing power and improve user task execution performance [20]. Assuming that multiple users can simultaneously offload their tasks to MEC through cellular links, each user can be allocated a particular amount of computing resources.

RETRACTED

The simulation scenario consists of a cellular MEC system supporting dense networks composed of multiple small base stations and multiple users. The simulation area is 1000m×1000m. The users and small base stations are randomly distributed in the simulation area. The simulation parameters are shown in Table 2. The task input data volume, the number of computing resources required to complete the task, the user’s computing power, the base station bandwidth and access capability, and the MEC server’s computing power and service capability are chosen to describe the difference between task requirements, user equipment, small base station access capabilities, and MEC server service capabilities [21].

**Table 2:** Simulation parameter determination of the multi-hybrid intelligent algorithm model.

Parameter	Letter	Value	Parameter	Letter	Value
Number of small base stations	*M*	10	MEC server’s computing power	*F*_*j*_^*b*^	10 ~ 15 Gcycles/s
Number of users	*N*	20	The maximum number of users that the MEC server can serve	*S*_*i*_	3 ~ 5
The maximum number of users that can be connected to a small base station	*B*_*j*_	10 ~ 15 MHz	Task input data volume	*I*_*i*_	1 ~ 2 Mbits
Noise power	*ϭ*^*2*^	3–5	The number of computing resources required to complete the task	*E*_*i*_	0.5 ~ 0.6 Gcycles
The number of computing resources required to complete the task	*D*_*i*_	-75 dBm	User’s computing power	*F*_*i*_	1 ~ 2 Gcycles

## 3. Results and discussions

### 3.1 Performance comparison of multi-stage-based task resource allocation model

Fig 5 shows the relationship between the number of tasks and the effect of data execution under different noise powers. As the amount of data transmitted by characters increases, the overhead of system task execution increases because the increase in the amount of input data leads to an increase in the time delay of task execution. Consequently, it leads to an increase in task energy consumption and further increases in overhead. Comparing the different noise powers in the proposed algorithm reveals that as the noise power decreases, the task execution overhead decreases; the algorithm in the literature has reached the same conclusion. Comparing the differences between different algorithms suggests that the proposed model’s task execution cost based on multi-stage portfolio server deployment is significantly lower than the literature algorithm. The reason is that the algorithm proposed in the literature aims to optimize the task execution delay. If the system’s processing efficiency is improved, more system computing power will be consumed, and the system’s energy consumption may increase, thereby causing the task execution overhead to increase.

RETRACTED

**Fig 5:** Th relationship between task execution overhead and task input data volume (different noise powers). Note: TD represents the proposed algorithm, and TM represents the algorithm mentioned in the literature.

Fig 6 shows the relationship between the number of tasks and the effect of data execution under different sending powers. As the amount of task transmission data increases, the system task execution overhead keeps increasing. However, the rate of increase in task overhead is lower than that of data under different powers. As far as the proposed algorithm is concerned, with the increase in sending power, the task execution overhead also decreases. This is because increasing sending power can improve the transmission performance between the server and the base station, thereby further reducing the task transmission time delay. The task execution energy consumption increases with the increase in sending power. Compared with the algorithm mentioned in the literature, the proposed algorithm model’s task execution overhead and energy consumption are reduced. However, the reduction is not very large because of the slight increase in energy consumption caused by the small increase in sending power compared with the time delay under the current parameter settings. Therefore, with the increase in sending power, task execution overhead shows a downward trend.

**Fig 6:** The relationship between task execution overhead and task input data volume (different sending powers).

Fig 7 presents the relationship between task execution overhead and the MEC server’s computing capacity. As the MEC server’s computing power increases, the system’s task execution overhead continues to decrease. When the base station number is 5, the base station bandwidth increases, causing the task execution overhead to decrease. This is because the increase in base station bandwidth allows more data to be calculated, increasing task execution efficiency and reducing overhead. When the base station bandwidth is 10MHz, as the number of base stations increases, the system’s task execution overhead is significantly reduced, which is much lower than the reduction of different base station bandwidth and is similar to the reason for base station bandwidth. Changes in the number of base stations are far greater than the changes in base station bandwidth. Compared with the algorithm model mentioned in the literature, the proposed model can significantly reduce task execution overhead and energy consumption, decreasing as the MEC server’s computing power increases. This is because increasing the MEC server’s computing power can improve task execution performance and reduce task execution overhead. Increasing the number and the bandwidth resources of base stations can reduce task execution overhead and improve task offloading performance.

RETRACTED

**Fig 7:** The relationship between task execution overhead and MEC server’s computing power.

Fig 8 shows the relationship between task execution overhead and the number of requested users. As the number of requested users increases, the system task execution overhead continues to increase. This is due to the increase in users, which leads to a continuous increase in the amount of data for calculations. The proposed algorithm model is compared with the method mentioned in the literature. Results show that the proposed model can reduce task energy consumption and has the best effect. Both the ERA algorithm and the ORA algorithm have huge task execution overhead. In addition, the ORA algorithm consumes the most energy. When resource allocations increase, resource competition at the MEC server will cause system performance degradation.

**Fig 8:** The relationship between task execution overhead and the number of requested users. Note: TD represents the proposed algorithm, TM represents the algorithm mentioned in the literature, ORA denotes the Optimal Resource Allocation algorithm, and ERA denotes the Equal Resource Allocation algorithm.

Fig 9 illustrates the relationship between task execution time delay or weighted energy consumption and the number of requested users. As the number of requested users increases, the task execution time delay continues to increase. Comparing different time delays finds that the two have a big difference. Especially when the number of users is 15, the gap between the two is increasing. As the number of users increases, the time delay between the two is increasing. Various weighted energy consumptions are compared. When the number of users is 10, the difference between the two keeps increasing. As the number of users increases, the weighted energy consumption between the two is also increasing. The reason for such a situation is that the algorithm mentioned in the literature only optimizes task execution time delay under the constraint of energy consumption. The algorithm proposed here considers both task execution time delay and weighted energy consumption. It jointly optimizes task offloading and resource allocation strategies, which can compromise time delay and energy consumption.

**Fig 9:** The relationship between task execution time delay or weighted energy consumption and the number of requesting users.

RETRACTED

### 3.2 Performance comparison of multi-hybrid intelligent algorithm based on energy consumption optimization

Fig 10 displays the relationship between the task execution energy consumption and the number of algorithm iterations. As the number of iterations increases, the task execution energy consumption decreases in the proposed algorithm. However, the task-free offloading (RTU) algorithm and the random offloading algorithm do not change with the number of iterations. The reason is that the RTU algorithm and the random offloading algorithm are both non-iterative algorithms. Hence, their task execution energy consumption does not change with the number of iterations. Comparing different channels’ noise power finds that as the noise power decreases, the task execution energy consumption also decreases. This is because channel noise reduction will increase user transmission rate, which, in turn, reduces task execution time delay and task execution energy consumption. However, when the number of iterations is 6, all algorithms tend to be stable.

**Fig 10:** The relationship between task execution energy consumption and the number of algorithm iterations. Note: TD represents the proposed algorithm, TM represents the algorithm mentioned in the literature, RTU denotes the task-free offloading algorithm, and the server is the random offloading algorithm.

Fig 11 exhibits the relationship between task execution energy consumption and the task input data volume. As the number of input tasks increases, the task execution energy consumption continues to increase. This is because the increased task input data volume will increase the task execution time delay, leading to increased task execution energy consumption. When the required minimum task transmission rate is fixed, a comparison of different algorithm models finds that the proposed algorithm model has the best performance. In contrast, the random offloading algorithm performs the worst. When the algorithm is fixed, as the required minimum transmission rate increases, the required sending power increases, thereby consuming more task execution energy.

**Fig 11:** The relationship between task execution energy consumption and task input data volume.

Fig 12 displays the relationship between the task execution energy consumption and the number of computing resources required to complete the task. As the number of computing resources required to complete the task keeps increasing, the task execution energy consumption also increases. The reason is that dense computing tasks will increase execution time delay, thereby consuming more energy. Besides, different algorithms are compared. The results suggest that the RTU algorithm has the highest energy consumption, while the proposed multi-hybrid intelligent algorithm based on energy consumption optimization has the lowest energy consumption. This is because the random offloading algorithm only supports random task offloading rather than optimizing itself according to the number of computing resources required to complete the task. The algorithm mentioned in the literature fails to consider the fairness of task execution, resulting in excessive energy consumption for user tasks with poor transmission performance.

RETRACTED

**Fig 12:** The relationship between energy consumption and the number of computing resources required to complete the task.

Fig 13 illustrates the relationship between task execution energy consumption and the number of computing resources required to complete the task. The RTU algorithm has the highest task execution energy consumption among the four algorithms under the best and worst cases. The random task offloading algorithm’s energy consumption in the best case is lower than that of the RTU algorithm, indicating that task offloading has the advantage of saving equipment energy consumption. However, because the random task offloading algorithm fails to determine a combined strategy based on the channel gain between the user and the small base station and the MEC server’s load, its worst-case task execution energy consumption is close to that of the RTU algorithm. Besides, the task execution energy consumption announced in the literature is lower than the proposed algorithm’s energy consumption in the best case.

**Fig 13:** The relationship between energy consumption and the number of computing resources required to complete the task.

Nevertheless, the proposed algorithm’s energy consumption difference in the two cases is slight, with good fairness. The reason is that the literature focuses on the energy consumption of system task execution and optimizes task offloading and resource allocation strategies but fails to consider user fairness. Consequently, the energy consumption of user task execution is higher than the energy consumption obtained by the proposed algorithm.

### 3.3 Comparison and analysis of model performance in different situations

As shown in Fig 14, each algorithm’s performance differences are illustrated when the data in the area are uniformly distributed. Literature [22] proposed EdgeABC, an emerging Internet of Things architecture, introduced blockchain to ensure the integrity of resource transaction data and the profit of service providers and proposed task shunting and resource allocation algorithms. Literature [23] offloaded the MEC server’s calculation through the small cell base station, connected to the macro BS through the wireless backhaul, and shared the MEC server’s computing resources among the offloaded MUs. Literature [24] introduced the Lyapunov optimization theory to decompose the original problem into four separate sub-problems. These sub-problems were solved through decomposition methods and matching and used energy-saving computing and radio resource management to offload computing tasks online. In Fig 14A, the proposed algorithm achieves a greater throughput of training tasks. Specifically, compared with the literature [23] and the algorithm in literature [24], the training task throughput of the algorithm can be improved by 24% and 56%, respectively. In Fig 14B, the proposed algorithm has reached a higher resource utilization level than the algorithm in literature [23] and the algorithm in literature [24]. Compared with the literature [23] and the algorithm in literature [24], the system’s final resource utilization rates can be increased by 23% and 53%, respectively. The simulation results prove that since the algorithm in [23] and the algorithm in [24] separate the assignment of task data nodes and the allocation of resources, their final performance reflected in the throughput of training tasks is inferior to the proposed algorithm, and the average resource utilization of edge nodes is also worse. Similar results appear when the data conform to the normal distribution and the Pareto distribution.

RETRACTED

**Fig 14:** The performance difference of each algorithm when the data in the area are uniformly distributed.

Fig 15 shows the performance comparison of each algorithm when the data in the region conform to the normal distribution. Specifically, Fig 15A shows the performance comparison of the system training task throughput. Compared with the algorithm in literature [23], the systems training task throughput can be increased by 25%. Compared with the algorithm in literature [24], the system’s training task throughput can be increased by 50%. Fig 15B shows the performance comparison of system resource utilization. In this figure, compared with the algorithm in literature [23], the final resource utilization of the system is increased by 25%. Compared with the algorithm in literature [24], the resource utilization rate is increased by 62%.

**Fig 15:** The performance comparison of each algorithm when the data in the area conform to the normal distribution.

Fig 16 presents each algorithm’s performance differences in system training task throughput and system resource utilization when the data in the area conform to the Pareto distribution. According to the comparison of the system training task throughput given in Fig 16A, the system’s training task throughput can be improved by 23% and 46%, respectively, compared with the algorithm in literature [23] and the algorithm in literature [24]. Based on the comparison of system resource utilization rate given in Fig 16B, compared with the algorithm in literature [23], the system’s final resource utilization rate has increased by 23%. Compared with the algorithm in literature [24], the final system resource utilization has increased by 51%. In addition, when the data conform to Pareto distributed, even if the task throughput of the entire system is smaller than in other distribution modes, the resource utilization of the entire system is similar or even higher in the end. Because in the Pareto distribution, most data nodes have a larger amount of data than other distributions.

RETRACTED

**Fig 16:** The performance difference of each algorithm in system training task throughput and system resource utilization when the data in the area conform to the Pareto distribution.

## 4. Conclusion

A joint task offloading and resource allocation algorithm is proposed based on energy consumption optimization regarding server deployment in multiple portfolios. The maximum task execution energy consumption is defined as the maximum energy consumption required for each user’s task execution in the system. The constraints of task offloading, power allocation, transmission rate, and computing resource allocation are comprehensively considered. The joint task offloading and resource allocation problem is modeled as minimizing task execution’s maximum energy consumption. Since it is a problem of the machine learning algorithm, directly solving it with traditional optimization methods is difficult. A hybrid intelligent algorithm is proposed to convert the original problem into power allocation sub-problems, task offloading, and computing power allocation sub-problems. Moreover, the fractional planning method, variable relaxation, and substitution, and upper bound substitution methods are adopted to determine the joint task offloading and resource allocation strategy, thereby optimizing the user’s task execution energy consumption in the worst case in the system. The proposed model’s effectiveness is verified through comparisons with previous literature and traditional algorithms, which can reference the research on server optimization deployment.

There are several shortcomings. First, the performance of the model is analyzed under different conditions. All data are tested under mobile edge computing conditions; however, the cloud computing platform cannot implement simple data calculations and analyze the models’ performance under different computing powers. Second, the differences of different algorithms are analyzed under different conditions from a macro perspective. However, with the continuous development of algorithms, data mining or deep learning algorithms are not used for comparison and processing. In the future, static scenarios where the user’s location remains unchanged or the system remains static will be considered, and the user’s mobility and the dynamic characteristics of network resources can be further considered. Besides, if system resources change with time, how to predict the user’s possible task offloading behavior based on the user’s historical information to reserve corresponding resources for them and meet their task offloading requirements is worthy of further exploration. Secondly, the optimization goal is based on the task execution overhead of all users in the system and the largest execution delay of all entity tasks in the system. Moreover, the task offloading and resource allocation strategy is designed from a macro perspective, without considering users’ priority. Therefore, it is of great practical significance to study task offloading and resource allocation strategies based on user priority or task importance, formulate task offload priority criteria, and preempt offloading mechanism based on priority.

RETRACTED

## Supporting information

S1 Data (RAR)
